# *Lactobacillus helveticus* Prevents Periodontitis Induced by *Aggregatibacter actinomycetemcomitans* in Rats by Regulating *β*-Defensins

**DOI:** 10.1155/2022/4968016

**Published:** 2022-02-27

**Authors:** Ru Jia, Ronghua Shi, Danping Guan, Yubo Wu, Wenhao Qian

**Affiliations:** ^1^Department of Stomatology, Shanghai Xuhui District Dental Center, 500 Fenglin Road, Shanghai 200032, China; ^2^Department of Stomatology, Shuguang Hospital Affiliated to Shanghai University of Traditional Chinese Medicine, 201203, China

## Abstract

**Objective:**

To study the preventive effect of *Lactobacillus helveticus* (*L. helveticus*) on periodontitis induced by *Aggregatibacter actinomycetemcomitans* (*A. actinomycetemcomitans*) in rats.

**Methods:**

Eighteen 8-week-old female rats were randomly divided into three groups: Sham group, Trehalose group, and *L. helveticus* SBT2171 (LH2171) group. We measured the distance of the cementoenamel junction-alveolar bone crest (CEJ-ABC) to evaluate alveolar bone resorption. Hematoxylin-eosin staining was used to observe the histopathological changes of rat hemimaxillary tissues. We detected the expression of *β*-defensins, tumor necrosis factor-*α* (TNF-*α*), interleukin- (IL-) 1*β*, and IL-6 and the number of *A. actinomycetemcomitans* in rat gingival tissues by quantitative reverse transcriptase polymerase chain reaction. The levels of IL-1*β*, IL-6, and TNF-*α* in rat gingival tissues were also measured by enzyme-linked immunosorbent assay.

**Results:**

Compared with the Trehalose group, the distance of CEJ-ABC was prominently reduced and alveolar bone resorption was notably improved in the LH2171 group. And the infiltration of inflammatory cells in the hemimaxillary tissue decreased obviously, periodontal fibers were arranged neatly, connective tissue small blood vessels proliferated, and the number of *A. actinomycetemcomitans* reduced significantly in the LH2171 group. In addition, the mRNA expression and release of inflammatory factors in the gingival tissues in the LH2171 group were notably lower than those in the Trehalose group. On the 21st and 36th day, the expression of *β*-defensins in the gingival tissue of the LH2171 group increased significantly.

**Conclusion:**

*L. helveticus* improves alveolar bone resorption and increases the expression of *β*-defensins thereby inhibiting the number of *A. actinomycetemcomitans* and thus prevents periodontitis.

## 1. Introduction

Periodontitis is one of the most common oral diseases, which can easily lead to loose teeth or even loss of the affected teeth and periodontal redness, swelling, and bleeding [1, 2], which have a great impact on the quality of patients' life [3]. Moreover, the incidence of periodontitis is relatively high, with 35% of people over 30 years old and 80% of people over 65 years old suffering from periodontitis [4]. Some studies have shown that the incidence of periodontitis is bound up with the microbial environment in the oral cavity [5]. Although conventional oral cleaning treatment of periodontitis has a good effect at present, for the improvement of oral microorganisms, the effect is still not obvious and periodontitis is prone to recurrence after treatment [6]. Several studies have found that probiotics can effectively treat such oral diseases by improving the microbial environment in the oral cavity of periodontitis patients, such as *lactic acid bacteria* [7], *Lactobacillus rhamnosus* [8, 9], and *Lactobacillus reuteri* [10]. These probiotics can significantly lessen the expression of inflammatory factors tumor necrosis factor-*α* (TNF-*α*), interleukin- (IL-) 1*β*, IL-6, and IL-17A. In other words, the probiotics alleviate periodontitis by regulating the body's immune function.

*Lactobacillus helveticus* (*L. helveticus*) is a kind of lactic acid bacteria, which plays a prominent role in improving intestinal function. It has been found that *L. helveticus* has the peculiarity that modulates host immunity, including an increase in regulatory T cells and a decrease in inflammatory factors in rats [11]. Furthermore, *L. helveticus* can also prevent and treat collagen-induced arthritis by upregulating anti-inflammatory factors [12]. In recent years, *L. helveticus* has also been involved in the treatment of periodontitis. The study of Khasenbekova et al. [13] confirmed that the mass of probiotic containing *L. helveticus* can notably alleviate local inflammation in periodontitis. Kobatake et al. found that LH2171 can upregulate the expression of *β*-defensins in the oral cavity, thus improving periodontal disease caused by *Porphyromonas gingivalis* [14]. *Aggregatibacter actinomycetemcomitans* (*A. actinomycetemcomitans*) is a low-abundance Gram-negative oral pathogen that causes periodontitis and tooth loss in adolescents [15]. *A. actinomycetemcomitans* has been considered an important pathogen of periodontitis patients [16–18]. Studies have shown that *A. actinomycetemcomitans* can induce periodontal bone resorption through a variety of virulence factors [19]. At present, there is no literature reporting a related study of the effects of *L. helveticus* on *A. actinomycetemcomitans*-induced periodontitis. Therefore, in this study, we used *A. actinomycetemcomitans* to induce the construction of a rat periodontitis model to explore the preventive effect of *L. helveticus* on periodontitis, so as to provide a more theoretical basis for the clinical treatment of periodontitis.

## 2. Materials and Methods

### 2.1. Experimental Animal

Eighteen Sprague Dawley female rats of specific pathogen-free grade, aged 8 weeks and weighing 180-210 g, were provided by the Beijing Experimental Animal Research Center (Beijing, China). The animal feeding conditions were as follows: temperature: 22 ± 2°C, humidity: 40± 5%, light for 12 h, free access to drink and eat, and routinely fed for 1 week for experiments. This study was approved by the Ethics Committee of Shanghai Xuhui District Dental Center (2019-6) and conforms to the ethical standards formulated by the Chinese Medical Ethics Committee.

### 2.2. *L. helveticus* SBT2171 (LH2171) Preparation

LH2171 was obtained from Megmilk Snow Brand Co., Ltd (Tokyo, Japan). LH2171 was incubated in MRS broth (Difco, Detroit, MI, USA) for 16 h at 37°C and then centrifuged at 8000 × g for 10 min at 4°C. Subsequently it was washed twice with PBS and once with sterile distilled water and resuspended in 25% Trehalose solution. The suspensions were stored at -80°C for experimental use [14].

### 2.3. Periodontitis Model and Drug Treatment

Eighteen rats were randomly divided into three groups: Sham group, Trehalose group, and LH2171 group, with 6 rats in each group. For the Sham group, after 21 days of feeding, each rat was intragastrically fed with 1 mL of 5% Carboxyl Methyl Cellulose (CMC) once a day until the 35th day. For the Trehalose group, each rat was orally administrated with 2 mL of 25% Trehalose solution (Sigma-Aldrich) once a day for 35 days, and *A. actinomycetemcomitans* (HK1651, ATCC, Rockefeller, Maryland, USA) suspension (10^8^/CFU/mL of 5% CMC) was given orally from the 21st day, once a day for 14 days. For the LH2171 group, each rat was orally administered with LH2171 suspension (10^9^/CFU/2 mL), once a day for 35 days, and HK1651 suspension (10^8^/CFU/1 mL of 5% CMC) was given orally from the 21st day, once a day for 14 days. After the last oral administration of *A. actinomycetemcomitans*, the rats were routinely fed for 30 days and then sacrificed, and the maxillary, mandibular, and periodontal tissues were separated for index determination.

### 2.4. Alveolar Bone Resorption Determination

Alveolar bone resorption was measured with reference to the previous method [20]. The right maxilla of the rat was taken, and the gingiva was stripped. Hemimaxillary bone was stained with 1% methylene blue for 1 min at 25°C to distinguish the cement-enamel junction (CEJ). The buccal and lingual root surfaces of all molars were imaged with a digital camera. The vertical distance between the CEJ and the alveolar bone crest (ABC) was evaluated using ImageJ software to measure the distance in millimeters. The average of the 3 buccal and 3 lingual surfaces of each molar was calculated.

### 2.5. Hematoxylin-Eosin (H&E) Staining

Hemimaxillary tissues of rats in each group were collected and fixed with 4% paraformaldehyde. The fixed tissue was embedded in paraffin after decalcification. The embedded tissue sections (4 *μ*m) were dewaxed and then stained with hematoxylin for 5 minutes. After differentiation with hydrochloric acid alcohol and rinsing with tap water, the slices were stained by eosin for 30 s. After dehydrating in different concentrations of anhydrous ethanol and treating with xylene, the slices were transparently sealed with gum. The pathological condition of the hemimaxillary tissue was observed under a microscope, and the experiment was repeated three times.

### 2.6. Quantitative Reverse Transcriptase Polymerase Chain Reaction (qRT-PCR)

We collected the gingival tissues of rats and extracted the total RNA by a total RNA extraction kit (Invitrogen, Carlsbad, CA, USA) and determined the concentration and purity of it. Then, we synthesized cDNA by reverse transcription according to the instructions of the reverse transcription PCR kit (TaKaRa, Tokyo, Japan). The following parameters were used to perform qRT-PCR: 95°C for 1 min, 95°C for 40 s, 58°C for 40 s, 72°C for 45 s, performed 35 cycles, and 72°C for 10 min. *β*-Actin was used as internal control. The relative expression of the target gene was calculated by the 2^−*ΔΔ*Ct^ method. The sequence of primers used is shown in Table 1.

### 2.7. *A. actinomycetemcomitans* Determination

*A. actinomycetemcomitans* standard strain (ATCC43717) was purchased from ATCC (USA). Subgingival plaque of rats in each group was collected, and InstaGene Matrix kits (Bio-Rad, USA) were used to extract DNA from bacteria and samples. The conventional PCR product of *A. actinomycetemcomitans* was used as the target fragment to construct the recombinant plasmid containing the target gene of *A. actinomycetemcomitans*. The standard plasmids were continuously diluted, and then, qRT-PCR was performed to establish the standard curve. The samples to be tested were simultaneously subjected to qRT-PCR and compared with the standard curve to obtain the quantity of *A. actinomycetemcomitans*. The qRT-PCR system was based on Maeda et al.'s study [21].

### 2.8. Enzyme-Linked Immunosorbent Assay (ELISA)

IL-1 *β*, IL-6, and TNF-*α* ELISA kits (Nanjing Jiancheng Bioengineering Institute, Jiangsu, China) were used to detect the levels of IL-1 *β*, IL-6, and TNF- *α* in the gingival tissue. The detection steps were carried out strictly according to the instructions of the detection kit.

### 2.9. Statistical Analysis

The experimental data were statistically analyzed using SPSS 10.0 software. *T*-test was used for comparison between the two groups. The statistical significance of differences between groups was analyzed using one-way ANOVA and Bonferroni's multiple-comparison test. The results were expressed as mean ± standard deviation (SD). *P* < 0.05 was considered to indicate a significant difference.

## 3. Results

### 3.1. *L. helveticus* Improves Alveolar Bone Resorption Induced by *A. actinomycetemcomitans*

In order to evaluate the preventive effect of *L. helveticus* on periodontitis, we first tested its effect on periodontitis symptoms. The results showed that the distance from CEJ to ABC in the Trehalose group was significantly larger than that in the Sham group, while LH2171 could inhibit the increase of the distance from the CEJ to ABC induced by *A. actinomycetemcomitans*. The results indicated that *L. helveticus* can improve alveolar bone resorption (Figure 1).

### 3.2. *L. helveticus* Reduces the Injury of the Hemimaxillary Tissue in Rats with Periodontitis

The histopathological examination results of the hemimaxillary tissue of rats showed that in the Sham group, the gingival epithelium (including the conjunctival epithelium and sulcus epithelium) was intact, the periodontal ligament fibers were neatly arranged, and the alveolar bone was intact; in the Trehalose group, the epithelium was separated from the tooth surface, the epithelium proliferated to the root, the periodontal fibers were edematous and degenerated, and the inflammatory cell infiltration was observed; in the LH2171 group, inflammatory cell infiltration was obviously reduced, periodontal fibers were more neatly arranged, and connective tissue had proliferation of small blood vessels. These results showed that *L. helveticus* could attenuate damage to the hemimaxillary tissue of periodontitis (Figure 2).

### 3.3. *L. helveticus* Reduces the Number of *A. actinomycetemcomitans* in Subgingival Plaque of Periodontitis Rats

The effect of *L. helveticus* on the number of subgingival *A. actinomycetemcomitans* in rats with periodontitis was further detected. On the 65th day, *A. actinomycetemcomitans* in the gingival tissue of the Trehalose group and LH2171 group were detected. The result showed that compared with the Trehalose group, the number of *A. actinomycetemcomitans* in the LH2171 group was notably decreased (Figure 3).

### 3.4. *L. helveticus* Reduces the Levels of IL-1 *β*, IL-6, and TNF-*α* in the Gingival Tissue of Rats with Periodontitis

The inflammatory factors associated with periodontitis were further examined, and the results showed that the expression of IL-1 *β*, IL-6, and TNF- *α* in the gingival tissue of the Trehalose group increased obviously on the 36th and 65th day. But the expression of those in the LH2171 group was prominently lower than that in Trehalose group (Figures 4(a)–4(c)). In addition, the release of IL-1 *β*, IL-6, and TNF- *α* in the gingival tissue of the Trehalose group was also significantly raised, while the release of the factors in the gingival tissue of the LH2171 group was prominently lower than that of the Trehalose group (Figure 4(d)).

### 3.5. *L. helveticus* Decreases the Expression of the *β*-Defensin Gene in Gingival Tissues of Periodontitis Rats

To further investigate how *L. helveticus* prevents the development of periodontitis, we further examined the expression of *β*-defensin genes. The results showed that the expression level of *β*-defensins was significantly increased in the gingival tissues of the LH2171 group than the Trehalose group on the 21st day (*P* < 0.01). On the 36th day, the *β*-defensin expression in gingival tissues of both the Trehalose and LH2171 groups was significantly increased than that of the Sham group (*P* < 0.01). On the 65th day, the expression level of *β*-defensins was significantly reduced both in the Trehalose and LH2171 groups, and the expression level in the Trehalose group was significantly lower than that in the LH2171 group (Figure 5).

## 4. Discussion

The treatment of periodontitis has always been a difficult problem in clinical settings, but its specific pathogenesis is still unclear. A number of studies have shown that periodontitis may be caused by the deterioration of oral microbial environment due to some unhealthy living habits [22, 23]. Regulation of the oral microbial environment not only is good for periodontitis but also reduces the occurrence of distal diseases [24, 25]. Although oral cleansing can temporarily improve the microbial environment in the oral cavity, long-term treatment outcomes are not ideal due to poor compliance of patients after treatment [26]. Some studies have demonstrated that the microbial environment in the oral cavity can be effectively improved by *Lactobacillus reuteri* to achieve the purpose of treating periodontitis [9]. However, up to now, the price of *Lactobacillus reuteri* preparation in the domestic market is relatively high and it takes a long time, which is causing a greater economic burden to patients, so it is urgent to find an economical and effective treatment.

It has been shown that *Lactobacillus* can regulate barrier function and defensin production by inducing epithelial signal transduction and modulate inflammatory signaling [27]. In this study, we found that LH2171 could notably inhibit the increase of distance from the CEJ to ABC in rats caused by *A. actinomycetemcomitans* and reduce the inflammatory cell infiltration and the content of *A. actinomycetemcomitans* in subgingival plaque. These results indicate that *L. helveticus* can improve alveolar bone resorption and promote periodontal improvement in patients. This is consistent with the findings of Becirovic et al. [7]. *β*-Defensins are secreted by the epithelial tissues of the gingiva, oral mucosa, and salivary glands. As an important member of the defensin family, *β*-defensins are an antimicrobial peptide in the periodontal chemical barrier, which can directly kill pathogens or sterilize through chemical chemotaxis and synergistic action with lysozyme to control the homeostasis of the internal environment [28, 29]. *A. actinomycetemcomitans* is an important pathogen in periodontitis patients, which is highly expressed in gingival tissues of patients with periodontitis [30]. Some studies have suggested that *β*-defensins are low-expressed in the oral gingival epithelium of patients with periodontitis [31]. In this study, the expression of *β*-defensins in the periodontitis rat group did not differ from that in the Sham group at the 21st. However, after the oral administration of *L. helveticus*, the expression of *β*-defensins was significantly increased. At days 36 and 65, the expression of *β*-defensins in the gingival tissue of rats in the LH2171 group began to gradually decrease. These results indicate that *L. helveticus* is able to improve periodontitis by increasing the expression of *β*-defensins.

The level of inflammatory factors is the main index reflecting the severity of periodontitis. IL-1*β* is secreted by macrophages, monocytes, and other cells and participates in the inflammatory response of the body. TNF-*α* is an endogenous regulatory factor produced by the activation of monocytes-macrophages and T lymphocytes, which is involved in the chronic inflammatory activation in the development of periodontitis, resulting in periodontal tissue damage [32]. IL-6 is a powerful cellular chemokine, which can activate neutrophils and release a series of active products and then lead to local inflammation and which is significantly increased in patients with periodontal disease [33]. In this study, it was found that the expression levels of IL-1*β*, IL-6, and TNF-*α* in the gingival tissue of periodontitis rats were notably increased, while the oral administration of *L. helveticus* could inhibit the expression and release of inflammatory cytokines. Kobatake et al. [14] similarly demonstrated that LH2171 reduced the increase in proinflammatory cytokine expression in gingival epithelial cells induced by *Porphyromonas gingivalis* stimulation, which was associated with upregulation of *β*-defensin expression. This suggests that *L. helveticus* may inhibit the *A. actinomycetemcomitans*-induced inflammatory response in the rat periodontium through the upregulation of *β*-defensin expression. However, no specific experiments were conducted and the mechanism needs to be further investigated.

## 5. Conclusion

To sum up, *L. helveticus* can improve alveolar bone resorption and reduce inflammatory cell infiltration by increasing the expression of *β*-defensins and decreasing the number of *A. actinomycetemcomitans*, thus preventing periodontitis.

## Figures and Tables

**Figure 1:** The distance from the cement-enamel junction (CEJ) to the alveolar bone crest (ABC) in each group. Results are expressed as the means ± SD. ^∗^*P* < 0.05 and ^∗∗^*P* < 0.01*vs.* the Sham group. ^#^*P* < 0.05*vs.* the Trehalose group.

**Figure 2:** Histopathological changes of hemimaxillary tissues in rats of each group observed by H&E staining. Magnifications, 100x and 400x. Scale bar = 200 *μ*m. GE: gingival epithelium; PDL: periodontal ligament fibers; ALB: alveolar bone.

**Figure 3:** The expression of *A. actinomycetemcomitans* in the gingival tissue of rats in each group was detected by qRT-PCR. Results are expressed as the means ± SD of triplicate assays from three independent experiments. ^∗∗^*P* < 0.01*vs.* the Sham group. ^##^*P* < 0.01*vs.* the Trehalose group.

**Figure 4:** Expression and release of inflammatory factors in rats. (a) qRT-PCR was used to detect the expression level of IL-1*β* in the gingival tissues of rats on days 36 and 65 in each group; (b) qRT-PCR was used to detect the expression level of IL-6 in the gingival tissues of rats on days 36 and 65 in each group; (c) qRT-PCR was used to detect the expression level of TNF-*α* in the gingival tissues of rats on days 36 and 65 in each group; (d) ELISA was used to detect the release of IL-1*β*, IL-6, and TNF-*α* in the gingival tissues of rats in each group on day 65. Results are expressed as the means ± SD of triplicate assays from three independent experiments. ^∗∗^*P* < 0.01*vs.* the Sham group. ^##^*P* < 0.01*vs.* the Trehalose group.

**Figure 5:** The expression of *β*-defensins in the gingival tissue of rats in each group was detected by qRT-PCR. Results were expressed as the means ± SD of triplicate assays from three independent experiments. ^∗∗^*P* < 0.01*vs.* the Sham group. ^##^*P* < 0.01*vs.* the Trehalose group.

**Table 1:** qRT-PCR primer sequence.

Gene name	Primer sequence
*β*-Defensins	F: 5′-ACCGGAGAGTCTTCTCTTCCA-3′
	R: 5′-TCAGCCCGATGTGAAACGAT-3′

Aa	F: 5′-AGAGTTTGATCCTGGCTCAG-3′
	R: 5′-CACTTAAAGGTCCGCCTACGTGCC-3′

IL-1*β*	F: 5′-CCAGCTTCAAATCT CACAGCAG-3′
	R: 5′-CTTCTTTGGGTATTGCTTGG GATC-3′

IL-6	F: 5′-TCCAGTTGCCTTCTTGGGAC3′
	R: 5′-GTACTCCAGAAGACCAGAGG -3′

TNF-*α*	F: 5′- AGCCGATGGGTTGTACCT-3′
	R: 5′- TGAGTTGGTCCCCCTTCT-3′

*β*-Actin	F: 5′-CGAGCTGTCTTCCCATCCA-3′
	R: 5′-TCACCAACGTAGCTGTCTTTCTG-3′

## Data Availability

The data used to support the findings of this study are available from the corresponding author upon request.
